# Intervention Effect of Evidence-Based Nursing on Postoperative Recovery of Vacuum Sealing Drainage in Patients with High Perianal Abscess with Magnetic Resonance Imaging Sequence Images

**DOI:** 10.1155/2022/1405134

**Published:** 2022-06-24

**Authors:** Xiaoxia Chen, Qingzhu Tang, Hongbiao Luo, Xianghong Zhong

**Affiliations:** Department of Anorectal surgery, Chenzhou First People's Hospital, Chenzhou 423000, Hunan, China

## Abstract

The purpose of this study was to evaluate the intervention effect of evidence-based nursing (EBN) on vacuum sealing drainage (VSD) recovery of patients with high perianal abscess after vacuum sealing drainage based on magnetic resonance imaging (MRI) sequence images. 60 patients with high perianal abscess were selected, and 30 patients before VSD were selected as the control group. Routine nursing was implemented in the control group, 30 patients after VSD were observed, and EBN was implemented in the observation group. The detection rates of various types of perianal abscess with different sequence combinations were studied, and the effects of EBN on pain and anal function scores of perianal abscess patients were analyzed. Anal function and defecation were assessed, and postoperative complications were calculated. Different combinations of MRI sequences can reach higher detection rates of intersphincter abscess and ischial anal abscess. The observation group had better pain relief and anal function recovery. The complication rate of the observation group was 16.67%, which was significantly lower than that of the control group (*P* < 0.05). It was confirmed that different MRI sequence combinations had higher detection rates for intersphincter abscess and ischial fossa abscess. EBN can promote the recovery of anal function and reduce complications in patients with perianal abscess.

## 1. Introduction

Perianal abscess is an acute suppurative infection of the anal glands which develops into the perianal space through the anal gland duct to form an abscess, which is prone to form anal fistula after the abscess ruptures [1]. Traditional antibiotics can relieve the clinical symptoms of patients in the treatment of perianal abscesses, but cannot prevent the formation of pus and the expansion of the abscess cavity effectively [2]. Magnetic resonance imaging (MRI) is one of the most important examination methods for perianal abscesses. This has the advantages of noninvasive convenience and accurate results and is widely recognized by patients. In clinical medicine, MRI, an advanced medical imaging technology, has been widely used and has become an indispensable means of clinical diagnosis, treatment, and research [3]. However, the lesion area is mainly found by observing the two-dimensional image sequences, which needs to be judged by the doctor's experience to a certain extent. The combination of different MRI sequences can display the structure and characteristics of the lesions more comprehensively and intuitively, improving the detection rate and the accuracy of diagnosis.

The main cause of perianal abscess is anal gland infection. Incision and drainage are the key to cure. To ensure smooth drainage, the internal opening of the abscess must be left open to effectively prevent microbial invasion and reduce infection [4, 5]. The most effective and common method for clinical treatment of perianal abscess is surgery [6]. Vacuum sealing drainage (VSD) is common in the treatment of inflammatory diseases, with good therapeutic effect, so it has been rapidly promoted and applied in clinical practice [7]. In recent years, VSD has been widely used for large cavity drainage after thoracic surgery, abdominal surgery, and orthopaedic surgery as well as drainage of infected wounds. In particular, VSD has a great effect in the application of perianal abscess surgery, which can reduce tissue edema, promote blood circulation, avoid wound contamination, reduce the probability of infection, and promote early healing of the wound [8]. The disadvantage of VSD is that the optimal pressure value during treatment is not uniform, in which there is a randomness in clinical implementation. Poor control of the pressure value will affect the effect. If the negative pressure is too big, it will cause bleeding and pain in the patients. If the negative pressure is too small to fully drain, the coagulant substances in the secretions are easy to agglutinate and the drainage tube is prone to blockage. Appropriate negative pressure is an important condition to ensure the effect.

Evidence-based nursing (EBN) is a new nursing model that provides high-quality nursing care through problem-finding, observation, and active application [9]. For the EBN model, the nursing activities by nursing staff are arranged to formulate detailed and comprehensive plans, combining scientific research conclusions with clinical experience and patient needs, and certain conclusions are drawn as the basis for decision-making of clinical nursing. This process is an essential link in evidence-based medicine [10]. It has good application effect in various medical practices [11, 12]. EBN can not only improve the efficiency of daily nursing operations but also improve the quality of nursing, promote the recovery of patients, and relieve pain and negative emotions of patients, making patients get better comfort and satisfaction [13–15]. In recent years, EBN has developed rapidly and clinical nurses have gradually developed the evidence-based awareness, to carry out EBN practice one after another.

In this study, the effects of different MRI sequence combinations on the detection rates of various types of perianal abscesses were discussed. The pain, anal function, defecation, and complications of the two groups were compared, which provided guidance and reference for the nursing methods of patients with perianal abscess.

## 2. Materials and Methods

### 2.1. Research Objects

A total of 60 patients with high perianal abscess who received treatment in hospital from April 2020 to March 2022 were selected as the research object. Thirty patients before VSD were selected as the control group, including 18 males and 12 females, aged 18.43 to 49.75 years, with an average age of 31.78 ± 7.98 years. Thirty patients after VSD surgery were selected as the observation group and received EBN after surgery. In the observation group, there were 17 males and 13 females, aged between 18.22 and 50.17 years, with an average age of 31.12 ± 7.33 years. There was no statistical difference in the general data of patients between groups (*P* > 0.05), which indicated a comparability. This study was approved by the ethics committee of hospital, and all the enrolled patients were informed and consented.

The inclusion criteria were described as follows: all the patients met the relevant diagnostic criteria of *Ding's Coloproctology* accurately. All the patients and their families voluntarily signed the informed consent. Ultrasound of the rectal cavity showed the high abscess.

The exclusion criteria below were followed: the patients had systemic diseases or an allergic constitution; the patients were complicated with rectal and anal canal tumors, or inflammatory bowel diseases.

### 2.2. MRI Examination

A 1.5 T magnetic resonance scanner was used for image collection at 5–20 images per second using the Cartesian full sampling method. The collecting parameters were listed as follows: the time of repetition/time of echo was 155.35/1.04 ms, the field of view was 300 × 360 mm^2^, the flip angle was 52°, the slice thickness was 7 mm, the matrix dimension was 160 × 192, and the imaging time was 300 s. First, sagittal T2 weighted imaging (T2WI) was performed through the midline of the patient's body to determine the position of the anal canal. Then, coronal and axial scanning of the anal canal was performed in axial T1 weighted imaging (T1WI), T2WI, and fat-suppression T2WI (T2WI-FS); coronal T2WI and T2WI-FS; and sagittal T1WI and T2WI.

### 2.3. Methods

In the control group, routine nursing was adopted, the vital signs of patients were monitored, and the drainage tube was also regularly monitored to ensure the unobstruction of the tube. The color and properties of the drainage fluid were closely observed, and the drugs were administered as prescribed by the doctor.

In the observation group, the patients with perianal abscess were treated with EBN, which was carried out following the methods below:

1. Effective negative pressure was maintained. It was generally believed that the negative pressure value between 200 and 300 mmHg is more appropriate. Regular ward rounds were performed to check the dressing and drainage of VSD. It was observed whether the negative pressure value was normal, whether the VSD dressing was collapsed, and whether the drainage tube has a tube shape. The connection and sealing of the drainage tube and the drainage tube itself were also checked. Listening carefully if there was the hissing sound of air leakage, to exclude the occurrence of air leakage; the seal was reinforced with a semipermeable membrane if necessary.
2. For the drainage nursing, the vacuum connection tube should be fixed effectively to avoid discount and pressure. The patients were told to ensure the smooth drainage of the tube when turning over. The disposable negative pressure closed drainage bottle was replaced every day, the drainage fluid was >2/3, and it was checked whether the drainage bottle was damaged and whether the tube was cracked. When replacing the drainage bottle, the aseptic operation should be strictly performed. The negative pressure should be turned off first, and the drainage tube should be clamped with a hemostatic forceps. The tube was then separated, and the connection of drainage tube should be sterilized with 75% alcohol before reconnecting. The negative pressure was readjusted after the replacement, and it was observed whether the drainage was effective. The date and time of the replacement were marked. The fixed position of the drainage bottle should not be higher than the wound, so as to avoid retrograde infection. The color, character, and quantity of the drainage fluid were closely observed and recorded in the nursing record sheet in time on each shift. When the fresh blood was drained, it was suspected that there was a possibility of active bleeding and it should be reported to the doctor for treatment in time.
3. Pain care was conducted. Analgesia should be given according to the duration and property of pain in patients. VSD was propagated well, supplemented with the stories of successful cases to encourage patients to build up confidence.
4. For the psychological care, the patients were cared and comforted. The knowledge about perianal abscess and the influence of constipation on the body and postoperative incision were explained to the patients. Patients were instructed to take deep breaths during defecation to effectively relieve pain and eliminate their fear of defecation.
5. For the rehabilitation treatment, classroom explanation was carried out for health education, in which the etiology of perianal abscess, precautions during and after surgery, and postoperative complications were explained. A guide was given to patients to cultivate a healthy lifestyle and behavior. A diet plan was made on the basis of the patients' postoperative conditions. The patients were instructed to eat more high-fiber foods and avoid fishy, spicy, and stimulating foods. They were also asked to drink about 1000 mL water every day to ensure smooth defecation. They were encouraged to take movement in bed 12 hours after surgery to avoid abdominal distension and constipation caused by long-term bed rest. The importance of regular bowel movements was publicized to the patients to cultivate an awareness of regular bowel movements. The patients should focus on when defecation as distraction was prohibited, and they should not squat for a long time to avoid bleeding or edema. They should not also restrain and endure the urge to defecate, and for those who cannot defecate on their own, 20 mL Kaisailu glycerine enema could be injected into the anus to help defecation. If the stools were hard in the rectum, glycerin or soapy water enema could be utilized. According to the defecation situation of the patients, medicine could be taken as prescribed by the doctor, and the defecation situation after medication should be observed.

### 2.4. Observation Indicators

The detection rates of various types of perianal abscesses scanned by different sequence combinations were calculated. The sequence combinations mainly included axial T1WI + T2WI-FS, coronal T1WI + T2WI, coronal T1WI + T2WI-FS, axial T1WI + T2WI, and sagittal T1WI + T2WI. The main types of perianal abscesses were intersphincter abscesses, abscesses of ischioanal space, pelvic-rectal abscesses, and abscesses of rectal wall.

The visual analogue scale (VAS) was adopted for evaluating the pain degree of patients, with a score of 0–10. The higher the score, the more severe the pain.

The anal functions of patients were evaluated using the Wexner anal incontinence score, which ranged from 0–20 points. The higher the score, the worse the anal functions.

The pain scores of postoperative Verbal Rating Scale (VRS)-5 were compared, where 0 indicated no pain and 5 indicated the unbearable pain.

The anxiety of the two groups of patients was compared. The Self-Rating Anxiety Scale (SAS) was adopted for scoring the psychological status of the patients. Less than 50 points meant the patient had no anxiety, 50–59 points were assessed as mild anxiety, 60–69 points meant the moderate anxiety, and more than 70 points indicated severe anxiety. The lower the score, the better the psychological status of the patients.

The defecation situation of the patients was also recorded. It was scored as 0 for smooth defecation and self-defecating, 1 point for unsmooth defecation but without the aid of drugs, and 2 points for unsmooth defecation or defecation only with the aid of drugs.

The degree of edema, anal wetness, infection, anal fistula, and other complications of the patients were observed.

### 2.5. Statistical Methods

SPSS21.0 was used for statistical analysis of data. Measurement data were expressed in the form of mean ± standard deviation, and the measurement data between two groups were compared using independent samples *t*-test. Enumeration data were compared in the form of percentage (%), and the comparison between two groups was expressed using the chi-square test. *P* < 0.05 indicated that a difference was statistically significant.

## 3. Results

### 3.1. Comparison of Detection Rates of Different Sequence Combinations for Various Types of Perianal Abscesses

Figure 1 displays different MRI-sequence images of patient 1. The patient had a horseshoe-shaped abscess in the sphincter space and extended to the left sciatic-anal fossa.

### 3.2. Comparison of Detection Rate of Different Sequence Combinations for Various Perianal Abscesses

Figure 2 represents the detection rate of various types of perianal abscesses scanned by different sequence combinations, in which Figures 2(a)–2(d) show intersphincter abscess, abscess of ischioanal space, pelvic-rectal abscess, and rectal wall abscess, respectively. The detection rate of intersphincter abscess was relatively higher for each sequence combination, among which, the detection rate of T1WI + T2WI-FS in the axial position was the highest, reaching 96.88%. The detection rate of ischioanal abscesses was also relatively high, as that of axial T1WI + T2WI-FS, coronal T1WI + T2WI, coronal T1WI + T2WI-FS, and axial T1WI + T2WI reached 100%. Scanned by T1WI + T2WI in the coronal position, the detection rate of pelvic-rectal abscess was the highest (100%). Coronal T1WI + T2WI, coronal T1WI + T2WI-FS, and sagittal T1WI + T2WI gave a detection rate of 100% for abscess of rectal wall, and the detection rate of T1WI + T2WI-FS in the axial position was 0%.

### 3.3. Comparison of VAS, VRS-5, Wexner, and SAS Scores before and after Nursing

Figure 3 displays the comparison of the VAS score, VRS-5 score, Wexner score, and SAS score before and after nursing. Figures 3(a)–3(d) represent the score of VAS, VRS-5, Wexner, and SAS, respectively. After nursing, the scores of the four terms of patients were all decreased, among which the VAS score decreased the most. The decrease of the scores of these four items in the observation group was significantly greater than that in the control group, showing the differences of statistical significance (*P* < 0.05).

### 3.4. Comparison of Stool Scores between Two Groups after Nursing

Figure 4 shows the comparison of stool scores between the two groups after nursing. In the observation group, 77% of patients had a defecation score of 0 after nursing and 17% and 6% had defecation scores of 1 and 2, respectively. The proportion of patients with a defecation score of 0 was relatively higher in the observation group, which was significantly higher than that in the control group (*P* < 0.05).

### 3.5. Comparison of Postoperative Complications between Two Groups

The incidence of postnursing complications is shown in Figure 5. After nursing care, the number of patients with anal wetting was 1 in the observation group, and the incidence was 3.33%. There was 1 case of infection, with an incidence of 3.33%. Edema occurred in 2 cases (6.67%). Anal fistula was found in 1 case, and the incidence was 3.33%. The total incidence of complications in the observation group was 16.67%, which was significantly lower than that in the control group (*P* < 0.05).

## 4. Discussion

Perianal abscess is one of the common diseases in the department of anorectal surgery, which mainly occurs in young and middle-aged men of 20–40 years old; the main cause is the anal sinus anal gland infection [16–18]. Surgery is the most common and effective treatment for perianal abscesses [19]. According to the types and conditions of the abscess, there are various surgical options. The main methods of clinical treatment of perianal abscess include simple incision and drainage, disposable radical incision, thread-drawing therapy, and various drainage techniques [20, 21]. VSD is a new cut surface treatment method with a smaller incision, requiring only a small radial incision of 1-2 cm, which can significantly reduce the degree of pain in patients [22]. The approach of VSD is outside the sphincter or at the sphincter tendon, reducing the damage to the sphincter during surgery and protecting the anal function to the greatest extent. Continuous negative pressure can collapse the abscess cavity, which is beneficial to the closure of the abscess cavity and the healing of the wound, reducing the length of hospital stay and promoting early recovery of patients [23]. Xue et al. [24] explored the therapeutic effect of VSD on wound repair time and inflammation in patients with soft tissue trauma compared with the traditional treatment. They found that the wound cleaning time, wound healing time, and hospital stay of patients after VSD treatment were all higher than those in the conventional dressing group, with the differences statistically significant (*P* < 0.05). VSD has obvious therapeutic effect on patients with soft tissue wounds, which could effectively shorten the wound healing time and reduce inflammation-related indicators. MRI has been widely used in the diagnosis of perianal abscesses, with good diagnostic results and high patient acceptance. Yang et al. [18] studied the diagnosis and prognosis of perianal abscess by MRI under the multimodal feature fusion algorithm, from which MRI image feature analysis under the multimodal feature fusion algorithm had a higher diagnostic performance. It had a positive effect on improving the detection rate, detection accuracy, and disease classification of perianal abscesses.

The effect of MRI-sequence images in evaluating the postoperative recovery of VSD in patients with perianal abscess was explored, and the effect of EBN was also explored on the VAS score, VRS-5 score, Wexner score, and SAS score of patients with perianal abscess. The anal functions of the perianal abscess patients who received VSD were evaluated, the defecation situation was counted, and the incidence of various complications of the patients after EBN was also counted. The detection rate of intersphincter abscesses was the highest in the T1WI + T2WI-FS axial plane, which reached 96.88%. The T1WI + T2WI-FS axial plane, T1WI + T2WI coronal plane, T1WI + T2WI-FS coronal plane, and T1WI + T2WI axial plane had a 100% detection rate for abscess of ischioanal space. The detection rate of T1WI + T2WI in the coronal plane also reached 100% for the pelvic-rectal abscess. All the T1WI + T2WI coronal plane, T1WI + T2WI-FS coronal plane, and T1WI + T2WI sagittal plane had a 100% detection rate as well for abscess of rectal wall. After EBN, the patients' VAS score, VRS-5 score, Wexner score, and SAS score in the observation group decreased, and the decreases were greater than those in the control group. This suggested that the pain in patients was greatly relieved and anal functions were well recovered as EBN was given. The patients with a defecation score of 0 accounted for 77% after EBN, having a larger proportion than that in the control group after nursing (*P* < 0.05). Thus, EBN could help improve the defecation of patients more quickly. The incidence of all the complications was 16.67% in the observation group, notably lower than that in the control group (*P* < 0.05). It was proved that, under EBN, the complications in patients became significantly less. EBN could promote the early recovery of patients with perianal abscess and reduce the incidence of complications.

## 5. Conclusion

The MRI images showed a good effect on the evaluation of postoperative recovery of patients with perianal abscess. Different MRI sequence combinations have a higher detection rate of intersphincter abscess and ischioanal abscess. EBN was beneficial to reduce the VAS score, VRS-5 score, Wexner score, and SAS score of patients with perianal abscess. Therefore, EBN could relieve pain, improve anal function, promote defecation, and reduce the probability of complications in patients. It was worthy of clinical application. The shortcomings of this research lay in that the sample size was small, in which further verification was needed. The sample size could be increased in the future to investigate the effect of EBN on the quality of life of patients with perianal abscess.

## Figures and Tables

**Figure 1:** Different MRI-sequence images of the patient with perianal abscess. A is the image of T1WI, B is T2WI, C is DWI, and D is ADC (male, 44 years old).

**Figure 2:** Comparison of the detection rates of various types of perianal abscesses by different sequence combinations. (a) Intersphincter abscess, (b) abscess of ischioanal space, (c) pelvic-rectal abscess, and (d) rectal wall abscess.

**Figure 3:** Comparison of VAS score, VRS-5 score, Wexner score, and SAS score between the two groups before and after nursing. (a) VAS score, (b) VRS-5 score, (c) Wexner score, and (d) SAS score. ^*∗*^Compared to the data before nursing, (*P*) < 0.05. ^#^Compared with the control group, (*P*) < 0.05.

**Figure 4:** Comparison of defecation score between the two groups after nursing. (a) Observation group and (b) control group.

**Figure 5:** Comparison of postoperative complications between the two groups. ^#^Compared with the control group, (*P*) < 0.05.

## Data Availability

The data used to support the findings of this study are available from the corresponding author upon request.
